# Application of Esmolol to Control Heart Rate and Artificial Intelligence Reconstruction Analysis for Rapid Zero-Cooperation Emergency Coronary CTA

**DOI:** 10.1155/2022/7363589

**Published:** 2022-02-26

**Authors:** Chenfeng Ni, Lei Pei, Miaoping Zhou, Xiaolong He

**Affiliations:** Department of Radiology, The Quzhou Affiliated Hospital of Wenzhou Medical University, Quzhou People's Hospital, Quzhou, Zhejiang 324000, China

## Abstract

**Objective:**

To investigate a rapid and effective method for the examination of coronary CTA in emergency patients requiring coronary CTA examination, who have faster heart rate (≧80 bpm) or cannot cooperate with the examination due to the inability of breath holding at poor physical conditions.

**Methods:**

Before coronary CTA examination, with the ECG monitoring, intravenous injection of esmolol was given to achieve rapid heart rate reduction. Without the patient's cooperation, coronary CTA examination was then performed in a quick and effective manner using the 640-slice high-speed CT. The diagnosis report was obtained through the subsequent reconstruction analysis using artificial intelligence software.

**Conclusion:**

Esmolol injection can rapidly reduce the heart rate of normal people during exercise and at rest, and the steady blood concentration can be reached in 2 minutes. The half-life is about 5 minutes, with short duration and fewer side effects on patients. The diagnostic rate of coronary artery segment using (excellent + good) CTA image of the patients with esmolol and artificial intelligence analysis in the experimental group was 95.4%, while the diagnostic rate was 91.1% in the control group, and there was no significant statistical difference between the two groups (*P* > 0.05). Esmolol injection can rapidly reduce heart rate in patients with high heart rate, without holding breath or long-term preoperative preparation; the combination with the analysis of subsequent artificial intelligence reconstruction is a new method for rapid and effective coronary CTA examination in all patients.

## 1. Introduction

Coronary atherosclerotic heart disease is a heart disease caused by coronary atherosclerotic lesions, such as vascular stenosis or obstruction, myocardial ischemia, hypoxia, or necrosis. Today, with the continuous development of technology, the diagnostic value of non-invasive rapid coronary angiography (CCTA) has attracted more and more attention in clinical practice. However, cardiac coronary CTA usually needs the cooperation of patients in breath holding state to reduce the artifacts of respiratory movement. For patients with breath holding difficulties, coronary CTA is often difficult to complete smoothly, especially for patients with respiratory diseases, poor cardiopulmonary function, and unable to cooperate with breath holding. The image quality obtained by coronary CTA is poor or even unavailable, which brings great difficulties to clinical diagnosis and follow-up treatment. Some patients have to accept cardiac DSA again, which also brings huge economic pressure and mental burden. Patients with high heart rate suffer from heart disease. Can coronary CTA be performed under free breathing? Because the heart rate of most patients is not ideal, the heart rate is often uncontrollable under the combined action of tension, claustrophobia, and chest pain. In addition, some elderly patients are unable to communicate properly, and it is difficult to form a good examination atmosphere. At present, most coronary CTA examinations are performed by oral BetalocZoc to reduce the patient's heart rate and improve the success rate of coronary CTA examination [1]. However, in clinical practice, some patients with high basic heart rate have tolerance to Betaloc ZOK, and some emergency critical patients are unable to reduce the heart rate below 80 bpm in a short time before examination [2]. This situation leads to low success rate and poor image definition of coronary CTA. In this study, esmolol was used instead of Betaloc ZOK to quickly and safely reduce the heart rate of emergency patients [3] and ensure that even patients who failed to reach the target heart rate or cooperate with the examination can successfully complete the coronary CTA examination. At the same time, the application of artificial intelligence reconstruction analysis can further improve the speed and accuracy of coronary CTA and greatly shorten the examination by more than one hour. Therefore, this is a positive improvement on the traditional examination method.

## 2. Data and Methods

### 2.1. Study Subjects

Emergency patients with coronary artery disease requiring a rapid diagnostic assessment of cardiovascular conditions and having a target heart rate above 80 bpm were included, excluding asthma, third-degree atrioventricular block, and severe chronic obstructive pneumonia. A Toshiba Aquilion ONE 640 slice high-speed volume CT was used to perform rapid artificial intelligence analysis of coronary CTA examination.

### 2.2. Study Methods

Patients candidated for coronary CTA examination were randomly divided into two groups: experimental group (*n* = 30) and control group (*n* = 30). In the experimental group, a new examination method with esmolol to control heart rate and artificial intelligence analysis requiring zero cooperation was used. The control group was treated with traditional Betaloc breath holding test and artificial reconstruction analysis. Esmolol Hydrochloride Injection was intravenously infused via an indwelling venous catheter before the examination, and real-time ECG data were provided by ECG gating. When the patient's heart rate was reduced below the target heart rate (≤ 70 bpm), coronary CTA examination was subsequently performed as scheduled. In the control group, conventional examination method requiring breath holding and administration of Betaloc ZOK was used. Statistical analysis was performed to detect any difference between the new method and conventional method.

### 2.3. Medication Method

(1) Control group: sublingual metoprolol tartrate tablet (25 mg/tablet) was administered as the conventional method, and the dose was defined as per the instructions and the basal heart rate of patients before the examination—sublingual metoprolol tartrate tablet 25 mg (1 tablet) for patients with heart rate>70 bpm and ≤80 bpm; sublingual metoprolol tartrate tablet 50 mg (2 tablets) for patients with heart rate >80 bpm and ≤90 bpm; sublingual metoprolol tartrate tablet 75 mg (3 tablets) for patients with heart rates >90 bpm and ≤100 bpm; the maximum dose should not exceed 100 mg. (2) Experimental group: for patients with heart rate > 70 bpm and≤80 bpm, esmolol injection 0.1 g combined with saline 10 mL was given via slow intravenous infusion; for patients with heart rate > 80 bpm and < 100 bpm, esmolol hydrochloride injection 0.2 g combined with saline 20 mL was given via slow intravenous infusion, and the maximum dose should not exceed 5 mg/kg. Adverse reactions: most adverse reactions are mild and transient. The most significant adverse reaction was hypotension. In case of adverse reactions, stop the drug immediately and observe the clinical effect. Atropine can be given for bradycardia; asthma can be treated with receptor agonists or theophylline; patients with cardiac insufficiency can be treated with diuretics and digitalis; patients with shock can be treated with dopamine, dobutamine, isoproterenol, and amrinone.

### 2.4. Other Preparations

A small amount of food and water was available on the day of examination, avoiding the examination at fasting or satiating condition. All patients in the control group rested for 20–30 min in a quiet environment and received breathing training; all patients in the experimental group were reviewed to understand and exclude contraindications. All patients were informed of detailed instructions regarding the examination, including the purpose of the examination, the requirement of heart rate, the upper arm soreness and generalized fever reaction upon rapid infusion of contrast agent, and even unexpected risk of allergic reaction to contrast agent in a few cases and vascular rupture. Therefore, each patient had a comprehensive understanding of the examination process and potential problems, avoiding the increased heart rate and abnormal heart rhythm due to psychological factors such as tension and fear.

### 2.5. Scan Protocol

Prospective Scanning scheme: 640 slice high-speed volume CT (tonshiba aquilion one CT) was used for prospective ECG gated volume scanning. Detector collimation was 320 x 0.5 mm; speed was 0.275‐0.32 seconds (automatically adjusted according to heart rate); the tube voltage and tube current are adjusted according to body mass index (BMI) and body shape. The tube voltage is 100 kVp or 120 kVp, and the tube current is from 200mA to 700 mA. The number of cardiac cycles and the optimal phase image to be collected were determined according to the manufacturer's recommended protocol, with heart rates of 60–79 bpm and >80 bpm. Two and three heartbeats were collected, respectively, and the R-R interval at 20%–80% phase images was used. Contrast agent 50–60 mL was injected *via* the right antecubital vein at a flow rate of 5.0 mL/s, followed by the injection of saline 30 mL at the same flow rate. The intelligence trigger sweep was performed using Sure Start software, and the trigger circle was positioned at the descending aorta in the central slices of the scanner field. When the first trigger threshold was >100 HU, the patients in the control group were instructed to inhale and hold their breath, and when the second trigger threshold was >250 HU, the enhanced scanning was initiated. In the experimental group, no breath holding was required, and the image data were acquired through direct scanning when the trigger threshold reached 250 HU.

### 2.6. Image Reconstruction

In the control group, the raw data of each patient were input for editing reconstruction using HCR algorithm or MCR algorithm, respectively. In the HCR subgroup, the heartbeat data acquired at one heartbeat were used for data reconstruction, and in the MCR subgroup, all heartbeat data acquired were used for reconstruction. The reconstruction parameters are as follows: slice thickness 0.5 mm, slice interval 0.25 mm, and transmit the best phase image data to the image post-processing workstation (Vitrea FX 6.7.3, vitalexend). The images of volume rendering (VR), maximum intensity projection (MIP), multiplanar reconstruction (MPR), and curved plane reconstruction (CPR) were made by vascular analysis software. In the experimental group, the optimal phase image data were imported into the AI artificial intelligence analysis software CoronaryDoc from Shukun (Beijing) Network Technology Co., Ltd., which automatically generated the images required for the diagnosis such as cardiovascular VR, MIP, MPR, CPR, and so on.

### 2.7. Image Quality Analysis

Patients were selected in a double-blind, free, randomized order. Two senior radiologists who have been engaged in cardiovascular diagnosis for many years were responsible for the analysis of coronary artery image quality of patients in both groups according to the 15-segment method recommended by the American Heart Association. All coronary artery segments with a diameter of >1 mm were evaluated. The image quality score was defined as follows: 3 points—coronary artery images were excellent and clear, without artifacts; 2 points—coronary artery images were good, with a few artifacts, which can basically satisfy the diagnosis; 1 point—coronary artery images were poor, with serious artifacts, which cannot satisfy the diagnosis.

### 2.8. Statistical Method

Independent sample *t*-test was used to compare the heart rate, subjective scores of images, and the signal-to-noise ratio between experimental group and control group. *P* < 0.05 level indicated that the differences were statistically significant. The conformance of the diagnostic scores by two radiologists was analyzed by kappa analysis: *k* < 0.40 indicated poor conformance, 0.40 ≤*k* < 0.75 indicated fair conformance, and *k* ≥ 0.75 indicated good conformance. All statistical analyses were completed using SPSS 20.0 (SPSS, Chicago, IL, USA).

## 3. Results

### 3.1. The Rate of Heart Rate Reduction in the Study Group Was Significantly Faster than That in the Conventional Control Group

This difference is caused by esmolol injection, which is an ultra-high selective *β*1 adrenoceptor blocker that rapidly reduces and slows the heart rate [4]. With respect to the pharmacokinetics, the action of conventional metoprolol tartrate tablet reached the maximum at 1–2 h after administration and lasted for a long period. In contrast, intravenous infusion of esmolol injection produced a rapid action at 1–2 min and maintained steady-state plasma-drug concentration within 5 min, which shortened the preparation time for heart rate in patients who underwent coronary CTA before the examination; at the same time, the action of the drug lasted for a short period, and the inhibition of *β*1-adrenergic receptor basically disappeared at 10–20 min after the termination of intravenous injection, which reduced the continuing effect of the drug on the patient's cardiac function after the examination (as shown in Table 1 and Figure 1). Esmolol can be rapidly metabolized *in vivo* and premodinantly metabolized by the liver before it reaches the systemic circulation. Iohexol, contrast agent used for coronary CTA examination, is mainly excreted by the kidneys, so the use of esmolol alleviates the burden on the kidneys and improves the safety of the drug [5].

As shown in Table 2, the mean heart rate at scanning was 69.23 bpm in the experimental group and 73.60 bpm in the control group (*P* value = 0.515), without significant difference; the mean subjective mean score was 2.63 in the experimental group and 2.53 in the control group (*P* value = 0.886), without difference between experimental group and control group. The *P* value for noise and signal-to-noise ratio was 0.662 and 0.310, respectively, which showed no statistical significance. The score conformance *K* value was 0.883 in the experimental group and 0.777 in the control group, and the diagnostic scores were relatively conforming, and there was no significant difference between the experimental group and the control group in the examination image quality.

The image quality in VR, MIP, and CPR between experimental group and control group was similar. There was no significant difference in the CT value and signal-to-noise ratio of coronary vessels. The image quality of the experimental group met the diagnostic criteria.

## 4. Discussion

Conventional coronary CTA has slow examination speed, long preparation time, and high requirement for patients, and it requires breath holding in order to effectively reduce artifacts caused by respiratory movements during the scan. However, in practice, many patients will be easily stimulated by various external factors such as tension and fear, and their heart rate cannot be controlled to the optimal state for the examination. In particular, some critically ill patients with acute myocardial infarction have insufficient time for preparation and waiting. The combination of various undesirable factors such as high heart rate, poor breath holding, and chest pain will greatly confound the coronary CTA examination, and high heart rate will cause poor image quality or even failure to obtain effective and clear images. Therefore, when the patient is unable to cooperate, reducing the heart rate of the examined patient is the most direct and effective method and means to improve the success rate of the examination [6, 7]. In this study, the quality of coronary artery imaging in patients with slow heart rate could still meet the diagnostic requirements, even when they are breathing freely. The above results are attributable to the following [8]. (1) The relative flow velocity of coronary artery (6.4–29.3 mm/s) caused by the expiration of the diaphragm in the normal breathing state (10–20 bpm) is much lower than the relative flow velocity of coronary artery (22.4–108.6 mm/s) caused by the heartbeat itself, so the weight of the artifacts caused by free breathing is not high. (2) In future, CT may develop to higher speed wide-body detectors, which will continuously improve the temporal resolution and accordingly effectively reduce various motion artifacts.

Previously, some researchers have attempted to evaluate the feasibility of coronary CTA during free breathing using dual-source CT, where the heart rate is required to be controlled below 60 bpm [9, 10]. Another researcher has assessed free-breathing coronary CTA using 320-detector CT; however, the heart rate is also required to be below 75 bpm due to limitations of temporal resolution and other factors [10]. Thus, it is feasible to perform free-breathing coronary CTA in subjects with low heart rates, but there is no effective method of coronary CTA examination in subjects with high heart rates (≥80 bpm) who are unable to hold their breath during examination. In this study, there is no requirement for the heart rate of the examined patients, 25 patients in the experimental group have a heart rate of >80 bpm, and the maximum heart rate reaches 109 bpm. Moreover, all 30 patients in the experimental group have a subjective image score of >2.6 points, which is not significantly different from the control group in terms of image quality and is sufficient to meet the diagnostic criteria (as shown in Figure 2). Meanwhile, the lower heart rate greatly improves the success rate of coronary CTA, and for some patients with low heart rate, only a single heartbeat or a lesser range of phase image is needed to complete the acquisition of image data, which in turn reduces the radiation dose given to patients [9, 11, 12].

With the advancement of technology and the thriving development of artificial intelligence, AI technology is gradually getting involved in traditional medical field to provide doctors with a faster and more accurate treatment protocol. In this study, AI cardiovascular analysis software from Shukun (Beijing) Network Technology Co., Ltd., is applied, which can automatically reconstruct the images required for the diagnosis such as cardiovascular VR, MIP, MPR, and CPR, automatically label the names of blood vessels, detect the location of lesions, severity of stenosis, and other indicators for diagnostic reports(as shown in Figures 3 and 4), and extract and print the required image films within 10 min. The overall reconstruction and diagnosis can be completed within 10 min, which greatly shortens the examination time for emergency patients with coronary artery disease and provides the surgeons with a comprehensive diagnostic report within the window phase of cardiovascular intervention, thus saving precious time for patients.

## 5. Conclusions

This study shows that the application of esmolol to control heart rate combined with artificial intelligence reconstruction analysis for rapid zero-cooperation emergency coronary CTA will substantially improve the feasibility and suitability of coronary CTA in critical conditions and make up for the non-usability of CT examination for some non-cooperative patients. It also significantly shortens the examination time of coronary CTA and improves the success rate of the examination. The shortcoming of this examination technique is that the new method must use 256-row and high-speed wide-body detector CT, and although esmolol reduces the heart rate of the examined subjects, a lower-row CT examination still requires breath holding scanning to improve the image quality. Secondly, the full-scale application of artificial intelligence analysis software is demanding time and effort. However, esmolol injection, instead of conventional oral Betaloc ZOK, to reduce heart rate still deserves the promotion, and the success rate of coronary CTA examinations with low heart rate is indeed higher than that of CTA examinations with high heart rate. It also reduces the patient's preoperative preparation procedure and saves the time for subsequent treatment.

## Figures and Tables

**Figure 1:** The rate of heart rate reduction of basal heart rate, esmolol experimental group, and Betaloc ZOK control group.

**Figure 2:** The subjective score, signal-to-noise ratio, and conformance *K* value between experimental group and control group.

**Figure 3:** The image quality in VR, MIP, and CPR of experimental group.

**Figure 4:** The image quality in VR, MIP, and CPR of control group.

**Table 1:** The rate of heart rate reduction in the study group and conventional control group.

Time	5 min	30 min	60 min
Basal heart rate	91 ± 15	90 ± 16	93 ± 13
Esmolol experimental group	69 ± 3	85 ± 5	92 ± 8
Betaloc ZOK control group	90 ± 15	86 ± 6	73 ± 4

**Table 2:** The subjective score, signal-to-noise ratio, and conformance *K* value between experimental group and control group.

Group	Experimental group	Control group	*P* value
Heart rate at scanning	69.23	73.60	0.515
Subjective score	2.63	2.53	0.886
Noise	59.46	61.20	0.662
Signal-to-noise ratio	15.46	15.26	0.310
Conformance *K* value	0.883	0.777	

## Data Availability

The data used to support the findings of this study are available from the corresponding author upon request.
